The article "miR-183-5p suppressed the invasion and migration of HTR-8/SVneo trophoblast cells partly via targeting MMP-9 in preeclampsia" was published in 2020. Journal: Biosci Rep.

# miR-183-5p suppressed the invasion and migration of HTR-8/SVneo trophoblast cells partly via targeting MMP-9 in preeclampsia

**DOI:** 10.1042/BSR20192575

**Published:** 2020-06-04

**Authors:** Mingli Suo, Yanfei Sun, Hailan Yang, Jing Ji, Yinfang He, Liyuan Dong, Yuxian Wang, Yanli Zhang, Yingan Zhang, Min Hao

**Affiliations:** Department of Obstetrics and Gynecology, The First Hospital of Shanxi Medical University, Taiyuan 030001, China

**Keywords:** clinical diagnosis, invasion, migration, miR-183, MMP-9, Preeclampsia

## Abstract

Preeclampsia (PE), a common obstetrical disorder, is characterized by impaired migration and invasion abilities of trophoblastic cells. MicroRNA-183-5p (miR-183) was reported to regulate cell migration and invasion in various types of human cancers; however, its role in the pathogenesis of PE remains elusive. Herein, we investigated the role of miR-183 in HTR-8/SVneo trophoblast cells invasion and migration and explored the underlying mechanism. Our results showed that miR-183 was significantly up-regulated in placental tissues from pregnant women compared with that in normal pregnant women. Overexpression of miR-183 inhibited proliferation, migration and invasion, as well as induced apoptosis in HTR-8/SVneo cells. Otherwise, down-regulation of miR-183 achieved the opposite effects. Bioinformatics prediction and luciferase reporter assay confirmed that matrix metalloproteinase-9 (MMP-9) is a target of miR-183. In addition, MMP-9 expression was significantly down-regulated, and inversely correlated with the miR-183 level in placental tissues from pregnant women with severe PE. Down-regulation of MMP-9 suppressed the trophoblast cell invasion and migration, whereas overexpression of MMP-9 promoted cell invasion and migration in HTR-8/SVneo cells. More importantly, up-regulation of MMP-9 reversed the inhibitory effects of miR-183 on cell invasion and migration in trophoblast cells. Collectively, our findings suggested that miR-183 may play critical roles in the pathogenesis of PE and serve as a potential biomarker for severe PE.

## Introduction

Preeclampsia (PE) is a pregnancy-associated disorder, which affects 3–5% of pregnancies, and is characterized by hypertension and proteinuria, which develops after 20 weeks of gestation in women [1]. According to American College of Obstetricians and Gynecologists (ACOG), PE is categorized into mild and severe. Severe PE is categorized as severe if systolic blood pressure (BP) is 160 mmHg or higher, diastolic BP of 110 mmHg or higher in two random urine samples, with either evidence of mild proteinuria, or mild hypertension plus severe proteinuria [2]. Severe PE, whether mild or, can develop into eclampsia, maternal multiorgan damage and death [3]. Despite extensive efforts, the pathogenesis of the disease is not fully understood. During early pregnancy, excessive trophoblast cell apoptosis and superficial trophoblast invasion leading to insufficient spiral artery remodeling and placental hypoxia are associated in the pathogenesis of PE [4,5]. Many molecular mechanisms have been revealed, but the role of microRNAs (miRNAs) in the trophoblast dysfunction seen in PE remains to be elucidated.

miRNAs are a recently discovered non-coding small RNAs (21–23 nucleotides), which negatively regulate gene expression at the post-transcriptional level via suppressing translation or inducing mRNA degradation [6,7]. Growing evidence indicates that these miRNAs play key roles in a wide variety of biological processes including cell proliferation, apoptosis, differentiation and migration [8]. Recent studies reported that an increasing number of miRNAs are found to be differentially expressed in placenta [9,10], indicating their potential role in the pathogenesis of PE. Furthermore, some studies revealed that miRNAs influence different aspects of trophoblast cells, such as proliferation, apoptosis, migration and invasion [11–13]. Notably, microRNA-183-5p (miR-183), a member of the miR-183-96-182 cluster located at the 7q31-34 locus of human chromosome, has been identified as an important regulator to suppress cell invasion in various types of cancers [14–16]; limited evidence demonstrated that miR-183 may involve in the development of PE. For example, Li et al. have documented that miR-183 is overexpressed in serum from PE patients and serves as a potential biomarker for PE [17]. However, the knowledge about the role of miR-183 in the pathogenesis of PE remains unclear.

In the present study, we compared the placenta miRNA expression profiles in placental tissues from pregnant women with PE and normal pregnant women using miRNA microarray, and miR-183 was selected for further study. Moreover, we explored the functions and molecular mechanism of miR-183 in the invasion of the trophoblast cells. Taken together, our results provide a theoretic basis for miR-183 as a predictive and therapeutic predictor for PE.

## Materials and methods

### Clinical samples

The human placentas (PE, *n*=30 and normal, *n*=30) were collected from women who underwent cesarean section at the Department of Gynecology and Obstetrics from June to December 2018 in the Department of Obstetrics and Gynecology, the First Hospital of Shanxi Medical University. The clinical characteristics of normal pregnant women and women with severe PE were shown in Table 1. Samples were immediately frozen in liquid nitrogen following delivery cesarean section and stored at −80°C until used. Placental tissues from normal pregnant women without PE or any other complications (premature rupture of membranes, maternal history of hypertension and/or renal or cardiac disease, fetal anomalies, maternal infection or smoking) were used as control [18]. Severe PE was defined as either severe hypertension (diastolic BP ≥ 110 mmHg) and mild proteinuria or mild hypertension and severe proteinuria (a 24-h urine sample containing 3.5 g protein or urine specimen ≥3+ protein by dipstick measurement) according to ACOG [2]. The research has been carried out in accordance with the World Medical Association Declaration of Helsinki, and all test subjects provided written informed consent prior to participating in the present study, which was approved by our university’s Institutional Review Board. All the procedures were approved by the Institutional Human Experiment and Ethics Committee of the First Hospital of Shanxi Medical University.

**Table 1:** Clinical characteristics of normal pregnant women and women with severe PE

Parameters	Control (*n*=30)	PE (*n*=30)	*P*-value
Maternal age at delivery (year)	26.4 ± 3.2	27.2 ± 4.1	0.7126
Nulliparous (%)	84.3	89.7	NA
Gestational age (weeks)	38.1 ± 4.2	34.6 ± 5.3	0.2631
Proteinuria (g/24 h)	Not detected	4.6 ± 3.4	NA
Systolic BP (mm Hg)	110.4 ± 17.2	165.7 ± 6.6	<0.01
Diastolic BP (mm Hg)	77.4 ± 4.5	104.2 ± 6.5	<0.01
Fetal birth weight (g)	3560.4 ± 513.9	2435.2 ± 501.7	<0.01

Abbreviation: NA, not available.

### Cell culture

Human trophoblast cell line HTR-8/SVneo was obtained from American Tissue Culture Collection (ATCC, Manassas, VA, U.S.A.) and maintained in RPMI-1640 medium (Gibco, Thermo Fisher Scientific, Waltham, U.S.A.) containing 10% fetal bovine serum (FBS, Invitrogen) and 1% penicillin/streptomycin (Sigma, St. Louis, MO) in a humidified incubator with 5% CO_2_ at 37°C.

### Cell transfection

The specific miR-183-5p mimics/inhibitor and corresponding negative control (NC) (mimics NC and inhibitor NC), as well as the siRNAs for matrix metalloproteinase-9 (MMP-9) (si-MMP9) and the respective scrambled siRNA (si-Scramble) were purchased from Ribobio (Guangzhou, China). The plasmid vector pcDNA-MMP9 and control vector pcDNA-vector were purchased from the BlueGene Biotech (Shanghai, China). These oligo-fragments were transfected into cells using Lipofectamine 2000 (Invitrogen, CA) according to the manufacturer’s protocol. The transfection efficiency was measured by real-time quantitative RT-PCR.

### miRNA microarray analysis

miRNA expression profiles were measured using miRNA microarray analysis. Total RNA was extracted from placental tissues using TRIzol reagent (Molecular Research Center, Inc., Cincinnati, OH, U.S.A.), and the miRNA fraction was further purified by an mirVana miRNA isolation kit (Ambion, Austin, TX) following the manufacturers’ guidelines. The isolated miRNAs were labeled with Hy3 using the miRCURY array labeling kit (Exiqon, Vedbaek, Denmark) and hybridized with miRCURY locked nucleic acid (LNA) microRNA arrays (v8.0; Exiqon). Replicated miRNAs were averaged, and miRNAs with intensities ≥ 50 in all samples were used to calculate a normalization factor. Expressed data were normalized by median normalization. Microarray images were taken with a Genepix 4000B scanner (Axon Instruments, Foster City, CA, U.S.A.) and analyzed with Genepix Pro 6.0 software (Axon Instruments).

### Quantitative real-time PCR

Total RNA was isolated from placental tissues or cells using TRIzol reagent (Molecular Research Center, Inc., Cincinnati, OH, U.S.A.) according to manufacturer’s protocols. The MMP9 and miRNA were reverse transcribed with TaqMan Gene Expression Assays kit and TaqMan MicroRNA Reverse Transcription kit (Applied Biosystems, Thermo Fisher Scientific, CA, U.S.A.), respectively. U6 was used as an internal control for miR-183, and GAPDH was used as an internal control for MMP-9. Real-time quantitative real-time PCR (qRT-PCR) was performed on an Applied Biosystems 7500 Real-Time PCR machine with miRNA-specific primers by TaqMan Gene Expression Assay (Applied Biosystems). The relative expression levels of miR-183-5p and MMP9 were calculated by using the 2^−ΔΔ*C*_t_^ method [19].

### Cell viability analysis

Cell proliferation was assessed using Cell counting Kit-8 (CCK-8) assay according to the manufacturer’s instructions [20]. Briefly, HTR-8/SVneo cells were seeded into 96-well plates and then transfected with matching oligonucleotides or plasmids. At 48 h after transfection, 10 μl CCK-8 reagent (1:10; Beyotime Biotechnology Co., Shanghai, China) was added for another 4 h culture at 37°C. The absorbance at 450 nm wavelength was used to evaluate cell proliferation. Each experiment was repeated three times.

### Apoptosis analysis

An annexin V-fluorescein isothiocyanate (FITC) (BD, Mountain View, CA, United States) and Propidium Iodide (PI, 50 μg/ml) (BD, Mountain View, CA, United States) staining were used to detect cell apoptosis according to the manufacturer’s instructions. HTR-8/SVneo cells were collected 48 h after transfection with their density adjusted to 1 × 10^6^/ml. Briefly, the cells were collected and washed twice with ice-cold PBS and then resuspended in binding buffer. The cells were then cultured with 5 μl Annexin V-FITC and 10 μl PI at room temperature in the dark for 20 min. Stained cells were analyzed using flow cytometry (BD, FACSCalibur, CA, United States). The measurements were performed independently for at least three times with similar results.

### Transwell cell invasion assay

Transwell assay was used to assess cell invasion *in vitro* 24 h after transfection. In brief, HTR-8/SVneo cells were seeded in upper chamber of Transwell chambers (8 μm pore size; Corning; Corning, NY, U.S.A.). The HTR-8/SVneo cells were seeded on the top side of the membrane precoated with Matrigel (BD, Franklin Lakes, NJ, U.S.A.). After 48 h of incubation, non-invading cells on the upper surface were carefully removed and invading cells on the lower surface of the membrane were fixed with methanol and stained with Hematoxylin (Solarbio). The cell numbers were counted from six random fields in each well at 200×. Experiments were performed in triplicate.

### Cell migration assay

The cell migration was evaluated using wound healing assay. The HTR-8/SVneo cells were plated on to six-well plates. After 48 h of incubation, and the migration status was examined by measuring the movement of cells into a scraped area created using a micropipette pipette tip. Images were taken at different points of time following wounding. The wound area was measured and the percentage of closure of denuded area was calculated by ImageJ software (NIH, Bethesda, MD, U.S.A.).

### Luciferase reporter assay

Partial sequences of MMP-9 3′-UTR containing miR-183 binding sites was amplified by PCR and cloned into the dual-luciferase reporter vector (pmirGLO; Promega, Madison, WI, U.S.A.) (wild-type pmirGLO-MMP-9-3′-UTR, wt). Mutation of the predicted binding site (mutation pmirGLO-MMP-9-mut-3′-UTR) was generated using the QuikChange Site-Directed Mutagenesis Kit (Stratagene, La Jolla, CA, U.S.A.) according to the manufacturer’s instructions. For the luciferase assay, the HTR-8/SVneo cells were grown in 96-well plates and co-transfected with 400 ng of either pmirGLO-MMP-9-3′-UTR or pmirGLO-MMP-9-mut-3′-UTR, and 50 ng miR-183 mimics/inhibitor or corresponding NC (Ribobio, Guangzhou, China) using Lipofectamine 2000 reagent (Invitrogen, CA). Forty-eight hours after transfection, the firefly luciferase activity was measured by dual-luciferase assays kit (Promega, WI) with *Renilla* luciferase activity as an internal control.

### Western blot analysis

The cells were lysed as described previously [21]. The protein concentration was measured using a BCA protein assay kit (Pierce, Rockford, IL). Protein samples (50 mg/sample) were separated by 10% SDS/PAGE gel (Sigma–Aldrich, St. Louis, MO) and then transferred to nitrocellulose membranes (Millipore, Bedford, MA, U.S.A.). Then, the membranes were blocked in 5% skimmed milk for 1 h at room temperature, and then incubated overnight at 4°C with primary antibodies against MMP-9 (Santa Cruz Biotechnology, Santa Cruz, CA, U.S.A.). β-actin (Sigma, St. Louis, MO, U.S.A.) served as an internal control. Then, the membranes were incubated with the horseradish peroxidase–conjugated (HRP) (Santa Cruz Biotechnology, Santa Cruz, CA, U.S.A.) secondary antibodies for 1 h at room temperature. Subsequently, the protein bands were scanned on the X-ray film using the enhanced chemiluminescence detection system (PerkinElmer Life and Analytical Sciences, Boston, MA). The measurements were performed independently for at least three times with similar results.

### Statistical analysis

All statistical analyses were performed using SPSS 14.0 software (Chicago, IL). Each experiment was repeated at least three times. Numerical data are presented as the means ± SD. When only two groups were compared, Student’s *t* test was conducted. One-way analysis of variance (ANOVA) followed by post-hoc tests were used to verify statistical differences among the groups. Correlation between mRNA and miRNA expression was analyzed with Spearman Rank correlation test. *P*-value of <0.05 was considered significant and <0.01 was considered to indicate a statistically significant difference.

## Results

### Clinical characteristics of normal pregnant women and women with severe PE

We first tested the clinical characteristics of the recruited pregnant women in the present study. As shown in Table 1, the systolic BP and diastolic BP in the women with severe PE were significantly greater as compared with the normal pregnant women (control group) (*P*<0.01). As compared with the control group, the fetal weight of women with severe PE was significantly decreased (*P*<0.01). There were no significant differences of the maternal and gestational age between normal pregnant women and women with severe PE (Table 1).

### miR-183 is up-regulated in the placental tissues from pregnant women with PE

To investigate the potential role of miRNAs in the pathogenesis of PE, a microarray assay was used in assess the miRNA expression profile in placental tissues from pregnant women with PE and normal pregnant women. As shown in Figure 1A, compared with control group, a large set of miRNAs were differently expressed, and miR-183 was one of the most significantly up-regulated miRNAs in placental tissues. To verify the expression trends of miR-183 obtained from microarray assay, we detected the miR-183 expression in the serum and placental tissues of normal and PE pregnancies using RT-qPCR assay. The results showed that miR-183 expression markedly up-regulated in the serum and placental tissues of PE pregnancies compared with that normal pregnancies (Figure 1B,C; *P*<0.01). Moreover, a dramatically positive correlation between miR-183 expression and proteinuria level was observed in PE pregnancies (r = 0.8030, *P*<0.01; Figure 1D). These results indicated that miR-183 may contribute to the progression and development of severe PE.

**Figure 1:** The expression levels of miR-183 in placental tissues and serum (**A**) The microarray analysis was used to identify the miRNA expression in the placental tissues from normal pregnant women and women with severe PE (*n*=3). Red or green color separately indicates high or low expression in the heatmap. (**B**) miR-183 expression in serum from PE and control group (*n*=30) were detected using qRT-PCR. (**C**) miR-183 expression was determined in placental tissues from PE and control group (*n*=30) by qRT-PCR. (**D**) The positive correlation between miR-183 expression and proteinuria level in PE pregnancies (r = 0.8030, *P*<0.01). Data are presented as means ± SD of three individual experiments.

### Overexpression of miR-183 inhibits HTR-8/SVneo cell migration and invasion

To explore the biological function of miR-183 in PE, we performed gain-of-function experiments by transfecting miR-183 mimics and performed loss-of-function experiments by transfecting miR-183 inhibitor into HTR-8/SVneo cells. RT-qPCR analysis confirmed that the expression of miR-183 was significantly up-regulated by miR-183 mimics transfection or down-regulated by miR-183 inhibitor (Figure 2A) (*P*<0.01). We then detected the role of miR-183 in regulating the proliferation, apoptosis and invasion of trophoblast cells. The results showed that overexpression of miR-183 markedly repressed cell proliferation, promoted apoptosis and inhibited the invasive and migratory abilities of HTR-8/SVneo cells, while miR-183 down-regulation exhibited opposite effects (Figure 2B–G). These results indicated that overexpression of miR-183 suppressed cell growth, migration and invasion in HTR-8/SVneo cells.

**Figure 2:** Effects of miR-183 on the cell proliferation, apoptosis, invasion and migration in HTR-8/SVeno cells The HTR-8/SVneo cells were transfected with miR-183 mimics/inhibitor or corresponding NC. (**A**) miR-183 expression was detected by qRT-PCR. (**B**) Cell proliferation was evaluated using CCK-8 assay. (**C**) Cell apoptosis was determined by annexin V-FITC/PI staining assay. (**D,E**) Cell invasion was assessed using transwell invasion assay. (**F,G**) Cell migration was measured by wound healing assay. Data are presented as means ± SD of three individual experiments (**P<0.01 vs. mimics NC, ^#^*P*<0.05, ^##^*P*<0.01 vs. inhibitor NC).

### miR-183 suppresses MMP-9 expression by directly targeting its 3′-UTR in HTR-8/SVneo cell

To investigate the target of miR-183 in HTR-8/SVneo cells, we performed the bioinformatics analysis (TargetScan 7.2) to predicate the putative targets of miR-183, and observed that MMP-9 is a potential target gene of miR-183 (Figure 3A). To verify this bioinformatics predication, we established the luciferase reporter plasmids containing the wt or mut 3′-UTR segments of MMP-9 (Figure 3A). Luciferase reporter assay showed that miR-183 mimics significantly reduced the luciferase activity in cells transfected with pmirGLO-MMP-9-3′-UTR when compared with mimic NC, whereas miR-183 inhibitor significantly enhanced the luciferase activity (*P*<0.01; Figure 3B). Additionally, miR-183 mimic/inhibitor did not affect the luciferase activity in the cells transfected with pmirGLO-MMP-9-mut-3′-UTR (Figure 3B). We next investigated whether miR-183 directly regulates the expression of MMP9 in trophoblast cells. We found that miR-183 overexpression significantly decreased the protein expression of MMP9, whereas miR-183 downregulation markedly promoted the expression of MMP9 in HTR-8/SVneo cells (Figure 3C). Moreover, our results demonstrated that the mRNA expression level of MMP-9 was dramatically decreased (Figure 3D), and was negatively correlated with miR-183 level in placental tissues from women with severe PE (r = −0.7658, *P*<0.01; Figure 3E). These data indicated that miR-183 suppress MMP-9 expression by targeting its 3′-UTR in PE.

**Figure 3:** MMP-9 is a direct target of miR-183 in HTR-8/SVeno cells (**A**) The MMP-9 3′-UTR region containing the wild-type (wt) or mutant (mut) binding site for miR-183. (**B**) The HTR-8/SVneo cells were co-transfected with either pmirGLO-MMP9-3′-UTR or pmirGLO-MMP9-mut-3′-UTR, and miR-183 mimic/inhibitor or corresponding NC and the relative luciferase activity were measured (**P<0.01 vs mimic NC. ^##^*P*<0.01 vs. inhibitor NC). (**C**) The HTR-8/SVneo cells were transfected with miR-183 mimic/inhibitor or corresponding NC, and the MMP-9 protein level was measured using Western blot analysis. β-actin was used as an internal control. (**D**) The MMP-9 mRNA level was detected using qRT-PCR in the placental tissues from normal pregnant women and women with severe PE (*n*=30) (**P<0.01 vs. control). (**E**) The negative correlation between MMP-9 and miR-183 levels in the in the placental tissues from women with severe PE (r = −0.7658, *P*<0.01). Data are presented as means ± SD of three individual experiments.

### The effects of MMP-9 on the HTR-8/SVneo cell invasion and migration

To investigate the role of MMP-9 in the invasion and migration of the HTR-8/SVneo cells, the cells were transfected with si-MMP-9/si-Scramble or pcDNA-MMP-9/pcDNA-vector. We first identified the efficiency of si-MMP-9 (si-MMP-9-1, si-MMP-9-2, si-MMP-9-3) against MMP-9 HTR-8/SVneo cells. As shown in Figure 4A, all three siRNAs significantly inhibited MMP-9 expression in HTR-8/SVneo cells compared with si-Scramble (*P*<0.01), and the siRNA (si-MMP-9-1) with the highest interference effect was chosen in subsequent experiments. In addition, transfection with si-MMP-9 or pcDNA-MMP-9 dramatically inhibited or increased the protein expression levels of MMP-9 in the HTR-8/SVneo cells compared with transfection with siRNA control or pcDNA-vector (*P*<0.01; Figure 4B,C). The *in vitro* functional assays (cell invasion and wound healing assays) demonstrated that knockdown of MMP-9 markedly suppressed cell invasion and migration compared with si-Scramble (*P*<0.01; Figure 4D,F). Conversely, overexpression of MMP-9 promoted cell invasion and migration compared with pcDNA-vector (*P*<0.01; Figure 4E,G). These results indicated that MMP-9 may act as an important regulator to modulate trophoblastic invasion in PE.

**Figure 4:** Effects of MMP-9 on the cell invasion and migration in HTR-8/SVeno cells The HTR-8/SVneo cells were transfected with si-MMP-9 and si-Scramble, or were transfected with pcDNA-MMP-9 and pcDNA-vector. (**A**) MMP-9 mRNA level was detected by qRT-PCR in HTR-8/SVneo cells transfected with si-MMP-9 and si-Scrambles (si-MMP-9-1, si-MMP-9-2, si-MMP-9-3). (**B,C**) MMP-9 protein expression was measured by Western blot analysis after transfection with si-MMP-9 or pcDNA-MMP-9. β-actin was used as an internal control. (**D,E**) Cell invasion was assessed using transwell invasion assay. (**F,G**) Cell migration was measured by wound healing assay. Data are presented as means ± SD of three individual experiments (**P<0.01 vs. si-Scramble; ^#^*P*<0.05,^##^*P*<0.01 vs. pcDNA-vector).

### Overexpression of MMP-9 rescues the inhibitory effects of miR-183 on HTR-8/SVneo cells

To validate whether miR-183 exerted the biological effect on trophoblast cells by targeting MMP9, HTR-8/SVneo cells were co-transfected with miR-183 mimics and pcDNA-MMP-9, and the cell proliferation, apoptosis, invasion and migration were assessed. As shown in Figure 5A,B, overexpression of miR-183 inhibits cell proliferation and promotes apoptosis in HTR-8/SVneo cells transfected with miR-183 mimics compared with control group (*P*<0.01), whereas up-regulation of MMP-9 reversed these effects of miR-183 on cell proliferation and apoptosis (*P*<0.01). Moreover, our results demonstrated that the suppressive effect of miR-183 on cell invasion and migration was partially rescued by overexpression of MMP-9 in HTR-8/SVneo cells (*P*<0.01; Figure 5C,D). These results suggested that miR-183 suppressed cell proliferation, invasion and migration by targeting MMP-9 in HTR-8/SVneo cell.

**Figure 5:** Restoration of MMP-9 aborts the suppressive effects of miR-183 on HTR-8/SVeno cells HTR-8/SVneo cells were transfected with miR-183 mimics or were co-transfected with miR-183 mimics and pcDNA-MMP-9/pcDNA-vector plasmid. (**A**) Cell proliferation was evaluated using CCK-8 assay. (**B**) Cell apoptosis was determined by annexin V-FITC/PI staining assay. (**C**) Cell invasion was assessed using transwell invasion assay. (**D**) Cell migration was measured by wound healing assay. Data are presented as means ± SD of three individual experiments (*P<0.05, **P<0.01 vs. control, ^##^*P*<0.01 vs. miR-183 mimics).

## Discussion

In the present study, we demonstrated that miR-183 was significantly up-regulated in the placental tissues from severe PE patients, and its expression was positively correlated with severity of proteinuria. The results indicated that elevated of miR-183 may be associated with the pathogenesis of PE. Overexpression of miR-183 suppressed cell proliferation, invasion and migration, and promoted apoptosis in HTR-8/SVneo cells. More importantly, our results further uncovered that miR-183 inhibited the invasion and migration of HTR-8/SVneo cells via targeting MMP-9 in HTR-8/SVneo cells.

Inadequate trophoblast invasion is so far recognized as the main cause for the development of PE [22,23]. Extravillous trophoblasts from fetal origin invade the uterine spiral arteries of the deciduas and myometrium in the early development of placenta, which can remodel of the placental vasculature and induce sufficient placental perfusion to nourish the fetus [24]. Recently, the miRNAs have been reported to be involved in the pathogenesis of PE, and play important role in the regulation of trophoblast cell invasion and migration, such as miR-210, miR-101 and miR-155 [25–27]. In the present study, we found that miR-183 level was significantly up-regulated in the serum and placental tissues of PE pregnancies, and its high expression was positively correlated the proteinuria level in PE pregnancies, indicating elevated of miR-183 may be associated with the pathogenesis of PE. Furthermore, up-regulation of miR-183 suppresses cell proliferation, invasion and migration, induces apoptosis in HTR-8/SVneo cells. These data suggested that miR-183 may act as an important regulator in the biological behaviors of HTR-8/SVneo cells.

MMP-9, a zinc-dependent proteinase, which involved in tissue remodeling, inflammation, processing of cytokines and mobilization of matrix-bound growth factors [28]. A previous study reported that MMP-9 levels were lower in the maternal serum samples from severe PE pregnant women than in the healthy controls, indicating that MMP-9 seem to be related to severe PE pathogenesis [29]. Several studies have demonstrated the involvement of MMP-9 in trophoblastic invasion and placentation [30–33]. Moreover, MMP-9 was identified to be involved in the invasiveness and metastasis of cervical cancer, as well as other malignant tumors including lung cancer, oseteosarcoma, renal cancer [34–36]. For example, Fan et al. have demonstrated that miR-183 inhibited cell invasion and metastasis in cervical cancer through targeting MMP-9 [37]. In this study, our results indicated that miR-183 suppressed MMP-9 level by targeting its 3′-UTR in HTR-8/SVneo cells. Meanwhile, MMP-9 expression level was dramatically decreased in placental tissues from women with severe PE, and was negatively correlated with the level of miR-183. Moreover, knockdown of MMP-9 inhibited cell invasion and migration in HTR-8/SVneo cells, whereas overexpression of MMP-9 promoted cell invasion and migration. More importantly, overexpression of MMP-9 partially reversed the inhibitory effects of miR-183 on cell growth and metastasis in HTR-8/SVneo cells. Taken together, these results indicated that miR-183 inhibited HTR-8/SVneo trophoblast cell invasion and migration by targeting MMP-9 in PE.

In summary, our results showed that miR-183 is up-regulated in the placental tissues from women with severe PE. miR-183 inhibited the invasion and migration of trophoblast cells via targeting MMP-9 partly. The data from present study suggested that miR-183 may play an important role in PE, and serve as a potential biomarker of severe PE clinical diagnosis.

## Abbreviations

ACOG: American College of Obstetricians and Gynecologists
BP: blood pressure
CCK-8: cell counting kit-8
FITC: fluorescein isothiocyanate
GAPDH: glyceraldehyde-3-phosphate dehydrogenase
miRNA: microRNA
miR-183: microRNA-183-5p
MMP-9: matrix metalloproteinase-9
PE: preeclampsia
PI: Propidium Iodide
RT-PCR: reverse transcriptase polymerase chain reaction
